The article "Application of Model-Building Based on Arterial Ultrasound Imaging Evaluation to Predict CHD Risk" was retracted in 2023. Reasons: signs of a paper mill; compromised peer review; unreliable results or conclusions.

# Application of Model-Building Based on Arterial Ultrasound Imaging Evaluation to Predict CHD Risk

**DOI:** 10.1155/2022/4615802

**Published:** 2022-09-19

**Authors:** Xiaoya Chen, Yinzhu Chu, Xiaobo Hou, Yue Han, Chunmei Zhang, Yue Zhang, Yue Leng, Changjun Wu

**Affiliations:** ^1^Department of Ultrasound, The First Affiliated Hospital of Harbin Medical University, Harbin, Heilongjiang 150001, China; ^2^College of Bioinformatics Science and Technology, Harbin Medical University, Harbin, Heilongjiang 150006, China

## Abstract

**Objective:**

Atherosclerotic is a chronic systemic disease that may occur in multiple vascular beds, including the carotid arteries, renal arteries, lower limb arteries, and cerebral vessels. Coronary atherosclerosis shares similar risk factors, pathogenesis, and pathophysiological basis with the atherosclerotic lesions of arteries at these sites. Arterial ultrasound assessment data were used to explore the correlation of atherosclerotic disease with CHD lesions and their severity and the number of lesion branches, as well as to evaluate its value in predicting CHD risk, in combination with traditional risk factors.

**Methods:**

A total of 363 inpatients with suspected CHD in the Department of Cardiology of the First Hospital of Harbin Medical University from November 2017 to June 2021 were selected. Patient clinical data, blood biochemical examination results, and ultrasound examination of neck vessels, abdominal arteries, and limb arteries were collected to obtain atherosclerosis assessment data. We then compared the differences between the CHD group and the control group, analyzed their correlation with CHD lesions and severity and the number of lesion branches, and evaluated the correlation with the coronary Gensini score. After adjustment for traditional risk factors, logistic regression was applied to analyze the relationship between arterial ultrasound assessment data and the risk of CHD. In addition, ROC plots were drawn to evaluate the risk of arterial ultrasound assessment data, combined with traditional risk factors, to predict CHD.

**Results:**

With regard to abnormal blood biochemical index values, differences in lipids, HDL-C, FIB, CK-MB, hs-cTnI, BNP, and GGT were found between the CHD group and the control group. Carotid plaque count, abdominal aortic flow velocity, inferior mesenteric artery flow velocity, classification of the number of stenotic branches of abdominal aortic branch arteries, lower-extremity-artery plaque count, degree of lower-extremity-artery stenosis, and lower-extremity-artery AS were risk factors for arterial ultrasound assessment data of CHD. Carotid plaque count, carotid artery AS, inferior mesenteric artery flow velocity, abdominal aortic flow velocity, abdominal aortic plaque count, abdominal aortic branch artery stenosis branch classification, lower-extremity-artery plaque count, lower-extremity-artery stenosis branch classification, degree of lower-extremity-artery stenosis, and lower-extremity-artery AS, combined with traditional risk factors, were mostly more effective than traditional risk factor models in predicting CHD, its severity, and the number of branch lesions; moreover, the predictive value was higher. Specifically, carotid plaque count, carotid AS, lower-extremity-artery AS, the degree of stenosis of lower-extremity arteries, and abdominal aortic branch artery stenosis branch classification can be used as predictor variables for CHD risk. Among these variables, the carotid plaque count can be used as an independent predictor of CHD.

**Conclusion:**

The incidence of arterial intima–media thickening (IMT), plaques, and stenosis can provide a reference for understanding the pattern of systemic atherogenesis and the distribution of atherosclerosis.

## 1. Introduction

Coronary heart disease (CHD) is a multifactorial coronary artery disease, characterized by high morbidity, mortality, and disability [1]. Coronary atherosclerosis shares similar risk factors, pathogenesis, and pathophysiological basis with peripheral atherosclerotic lesions and the abdominal aorta and its branches, allowing early CHD detection and the assessment of the risk of an acute attack of CHD individually with reference to the degree of atherosclerosis in other arteries [2, 3].

Ultrasound is a noninvasive, safe and quick, and easy screening tool that is inexpensive, easy to perform, and repeatable, rendering it suitable for widespread screening and universal access [4, 5]. Arterial ultrasound can observe the lesions of atherosclerosis, from typical lesions of early intimal thickening and plaque formation to arterial stenosis and even occlusion; moreover, the procedure is a noninvasive test to assess atherosclerosis [6–10].

The discovery of new predictors and correlative ultrasound indicators of CHD can provide new ideas for screening CHD in clinical patients and for medical authorities to develop guidelines for the prevention and intervention of CHD [11]. This can help improve the disease, reduce the occurrence of serious complications of CHD, reduce the disability rate, decrease the morbidity and mortality rates, promote the health of the entire population, and lower the burden on families and society.

In the current study, we performed ultrasound examinations of the carotid artery, vertebral artery, subclavian artery, abdominal aorta and its branch arteries, and arteries of the extremities in patients clinically diagnosed with CHD. We also observed the atherosclerotic lesion indices of each vessel, including intima-media thickening (IMT), plaque formation, presence of stenosis, number of stenotic branches, and degree of stenosis to understand the occurrence and distribution pattern of systemic atherosclerosis in the population. We screened the characteristic indices from arterial ultrasound to identify the independent predictors related to CHD. The correlation between CHD lesions, their severity, and the number of lesions was analyzed by combining the arterial ultrasound assessment of atherosclerotic indices, related clinical data, and blood biochemical indices. Finally, a stepwise logistic regression model was used to determine the optimal combination of arterial ultrasound assessment data and traditional risk factors to construct a CHD risk prediction model, increase the predictive value of risk scores, analyze their predictive efficacy, and improve the accuracy of the prediction model.

## 2. Materials and Methods

### 2.1. Study Subjects

A total of 363 patients hospitalized with suspected CHD in the Department of Cardiology of the First Hospital of Harbin Medical University from November 2017 to June 2021 were selected for CAG examination; on the basis of the CAG results, the patients were divided into the CHD group with 273 cases and the control group with 90 cases. Exclusion criteria were as follows: (1) patients with a combination of severe liver disease (e.g., coagulation disorders, ascites), severe renal disease (those with renal failure requiring dialysis), severe pulmonary disease (pulmonary heart disease, those with respiratory insufficiency, etc.), hematologic prodromes, autoimmune diseases, malignancies, or a history of psychiatric disorders; (2) persons with vascular diseases such as entrapment aneurysms of blood vessels, aortitis, arterio-venous fistulas of body vessels, thrombo-occlusive vasculitis, arterial myofibrillar dysplasia, and congenital arterial stenosis; (3) those with other cardiovascular diseases such as congenital heart disease, rheumatic heart disease, cardiomyopathy, and those with severe cardiac insufficiency; and (4) patients with previous vascular line reconstruction.

The patient was classified under the CHD group if stenosis diameter ≥50% in any of the following areas: the left main trunk, left anterior descending branch, left circumflex branch, right coronary artery, or major branch of the coronary artery. Meanwhile, a patient was classified under the control group if stenosis diameter <50%. The CHD group was further classified by the number of coronary artery lesions: single lesion, double lesion, and multiple lesions. The CHD group was further classified by the degree of severity of the most serious coronary artery: severe stenosis and occlusion. The study was approved by the Medical Ethics Committee (NO.2020169), and the study subjects signed an informed consent form.

### 2.2. Data Collection

General clinical information and the following blood biochemical indices of the patients were recorded: lipids (TC, TG, HDL-C, LDL-C, VLDL, ApoB), FIB, PLT, CK-MB, BNP, hs-cTnI, GGT, BUN, Cr, and UA.

### 2.3. Arterial Ultrasonography

Arterial ultrasound was performed using the Philips iE 33 or the Philips CX50 color Doppler ultrasound diagnostic instrument. During the examination, the subject was in a calm state and placed in a lying position, with the examination site fully exposed. The arteries of the whole body were then examined, including the carotid artery, vertebral artery, subclavian artery, upper limb arteries (axillary, brachial, ulnar, and radial arteries), abdominal aorta and its branches (including the celiac trunk, superior mesenteric artery, inferior mesenteric artery, and bilateral renal arteries), and lower limb arteries (femoral, popliteal, anterior tibial, and posterior tibial arteries).

### 2.4. Statistical Analysis

The data were statistically analyzed using SPSS 26.0 or Stata 14.0 or R statistical software, and the measurement data conformed to normality. For results expressed as mean ± standard deviation, a *t*-test was performed for comparison between the two groups. The measurement data were skewed and expressed as the median M (P25, P75), and the rank-sum test was performed for between-group comparison. Dichotomous or multicategorical data, expressed as percentages (%) (number of cases), were compared between the two groups by using the chi-square test or Fisher's exact test. Correlations between general clinical data, blood biochemical tests, and arterial ultrasound data that varied between the two groups, as well as the risk of CHD and severity and the number of lesion branches, were analyzed by binary logistic regression, expressed as OR values (95% confidence interval). Arterial ultrasound assessment data were correlated with the coronary Gensini score by Spearman correlation analysis for continuous data and Pearman correlation analysis for dichotomous or multicategorical data. After adjustment for traditional risk factors, logistic regression was applied to analyze the correlation of different arterial ultrasound assessment data with the risk of CHD lesions and their severity and the number of lesion branches, expressed as OR (95% confidence interval). *P* < 0.05 was considered statistically significant.

## 3. Results

### 3.1. Comparison of Baseline Characteristic Data between the CHD Group and the Control Group

This research included 363 participants consisting of 217 males and 146 females, with a mean age of (59.1 ± 9.7) y. They were divided into the CHD group with 273 patients and the control group with 90 patients on the basis of the CAG results. The CHD group consisted of 183 males and 90 females, with a mean age of (60.0 ± 9.6) y (age range: 84–33 y); the control group consisted of 34 males and 56 females, with a mean age of (56.4 ± 9.5) y (age range: 75–31 y). In the CHD group, 47 cases of single-branch lesions, 53 cases of double-branch lesions, 173 cases of multibranch lesions, 125 cases of severe stenosis, and 122 cases of occlusion were reported.

The CHD group and the control group varied in age, sex (male), height, history of diabetes, years of diabetes, diabetes typing, history of hypertension, maximum systolic blood pressure, history of smoking, years of smoking, number of cigarettes per day, total number of cigarettes smoked, years of alcohol consumption, and high-salt diet (*P* < 0.05).

### 3.2. Comparison of Blood Biochemical Indices between the CHD Group and the Control Group

With regard to the abnormal detection values of blood biochemical indices, significant differences in lipids, HDL-C, FIB, CK-MB, hs-cTnI, BNP, and GGT were found between the CHD group and the control group (*P* < 0.05, Table 1).

### 3.3. Comparison of Arterial Ultrasound Assessment Data between the CHD Group and the Control Group

Differences between the CHD group and the control group were found in the carotid artery internal diameter, subclavian artery flow velocity, brachial artery IMT, abdominal aortic internal diameter, abdominal aortic flow velocity, abdominal trunk flow velocity, superior mesenteric artery flow velocity, inferior mesenteric artery flow velocity, flow velocity and RI at the opening of the renal artery, RI at the hilar of the renal artery, and femoral artery IMT (*P* < 0.05, Figure 1, Table 2).

In addition, the results for IMT thickening and plaque showed differences in the number of carotid plaques, subclavian artery plaques, abdominal aortic plaques, and lower limb artery plaques (*P* < 0.05) and no differences in carotid IMT thickening and femoral artery IMT thickening (*P* > 0.05) between the CHD group and the control group.

For stenosis, significant differences between the CHD group and the control group were found in the carotid artery stenosis, number of stenotic branches, degree of stenosis and carotid artery AS, number of stenotic branches in the cervical vessels, abdominal trunk stenosis, superior mesenteric artery stenosis, number of stenotic branches in the branches of the abdominal aorta, lower-extremity-artery stenosis, number of stenotic branches, degree of stenosis, and lower-extremity-artery AS (*P* < 0.05).

### 3.4. Correlation Analysis of Arterial Ultrasound Assessment with CHD Lesions

We subsequently performed a binary logistic regression analysis for the data indicators that differed between the CHD group and the control group in arterial ultrasound. The following were found to be correlated with CHD lesions and their severity and the number of lesion branches: carotid artery internal diameter, subclavian artery flow velocity, abdominal aortic flow velocity, abdominal trunk flow velocity, inferior mesenteric artery flow velocity, carotid artery plaque count, lower-extremity-artery plaque count, abdominal trunk stenosis, abdominal aortic branch artery stenosis branch classification, branch classification of the stenosis of lower-extremity artery, and degree of stenosis of lower-extremity arteries (*P* < 0.05, Tables 3–8).

### 3.5. Correlation Analysis between Arterial Ultrasound Assessment and the Coronary Gensini Score

Subsequently, we conducted a correlation analysis for arterial ultrasound assessment and the coronary Gensini score. The following indicators were found to be positively correlated with the coronary Gensini score (*P* < 0.05, Table 9, Figure 2): carotid plaque count, carotid AS, submesenteric flow velocity, abdominal aortic plaque count, abdominal aortic branch artery stenosis branch count, lower-extremity-artery plaque count, lower-extremity-artery stenosis branch count classification, degree of stenosis of lower-extremity arteries, and lower-extremity-artery AS.

### 3.6. Diagnostic Value of Arterial Ultrasound Assessment for CHD

We then measured the diagnostic value of arterial ultrasound assessment for CHD by ROC curve analysis. The results are listed in Tables 10 and 11 and Figure 3.

### 3.7. Logistic Regression Analysis of the Predictive Value of Arterial Ultrasound Assessment and CHD Risk

After adjusting for traditional risk factors (clinical data and risk factors for blood biochemical indices), we performed a logistic regression analysis of the predictive value of arterial ultrasound assessment and CHD risk. The results showed that the following indicators were correlated with CHD lesions and their severity and the number of lesion branches (*P* < 0.05, Table 12): carotid plaque count, abdominal aortic flow velocity, inferior mesenteric artery flow velocity, the classification of the number of stenotic branches of abdominal aortic branch arteries, lower-extremity-arterial plaque count, the degree of stenosis of lower-extremity arteries, and lower-extremity-artery AS).

### 3.8. Predictive Model of the Diagnostic Efficacy of Arterial Ultrasound Assessment Combined with Traditional Risk Factors for Predicting CHD Risk and Its Severity and the Number of Lesion Branches

After adjustment for traditional risk factors (clinical data and risk factors for blood biochemical indicators), the AUCs of the carotid plaque count, carotid AS, inferior mesenteric artery flow velocity, abdominal aortic flow velocity, abdominal aortic plaque count, abdominal aortic branch artery stenosis branch classification, lower-extremity-artery plaque count, lower-extremity-artery stenosis branch classification, the degree of arterial stenosis in the lower extremities, and lower-extremity-artery AS combined with traditional risk factors in predicting CHD and its AUCs for severity and the number of lesions were markedly higher than those of traditional risk factor models.

The AUCs of the carotid artery plaque count for predicting the risk of CHD, severe coronary artery stenosis, and coronary artery occlusion were 0.901, 0.875, and 0.780, respectively; the AUCs of carotid artery AS for predicting the risk of CHD and the coronary artery single-branch lesion were 0.902 and 0.750, respectively; the AUC of lower-extremity-artery AS for predicting the risk of coronary artery occlusion was 0.798. The AUC of lower-extremity-artery stenosis for predicting the risk of coronary artery double lesion was 0.737; the AUC of branch abdominal aortic artery stenosis classification for predicting the risk of coronary artery multiple lesions was 0.802 (Figure 4).

## 4. Discussion

Atherosclerotic disease is currently considered a chronic systemic disease that can occur in multiple vascular beds, including the carotid, renal, lower-extremity arteries, and cerebral vessels [12–14]. Coronary atherosclerosis has similar risk factors, pathogenesis, and pathophysiological basis as atherosclerotic lesions of arteries at these sites. Ultrasound can examine carotid vessels, abdominal arteries, and extremity arteries to obtain atherosclerosis assessment data [15–17], explore its correlation with CHD lesions and their severity and the number of lesion branches, as well as evaluate its value in predicting CHD risk, in combination with traditional risk factors.

In the present study, we found a higher carotid plaque count and more carotid stenotic branches, more severe stenosis, and higher carotid AS in the CHD group. Numerous studies have recently shown a significant association between peripheral arterial plaque and CHD [18–20]. Polak et al. [21] showed that in multivariate corrected analysis, all plaque parameters were significantly associated with CHD incidence, with hazard ratios ranging from 1.27 to 1.80, with the strongest association for IMT >1.5 mm. We found that carotid plaque count was an independent factor influencing CHD in arterial ultrasound assessment and significantly varied between the case group and the control group (chi − squared value = 70.500 and *P* < 0.05). Binary logistic regression analysis indicated that the carotid plaque count was correlated with the severity of CHD lesions and the number of coronary artery lesion branches; moreover, the three plaque classifications were correlated with multiple coronary artery lesions (ORs: 2.449, 3.297, 5.680, *P* < 0.05).

The results of logistic regression analysis adjusted for traditional risk factors showed that the number of carotid plaques was correlated with the severity of CHD lesions and the number of lesion branches. Among them, (2 : 2) correlated with CHD, severe coronary artery stenosis, and multiple coronary artery lesions (ORs: 5.698, 5.534, and 3.215, respectively, *P* < 0.05); (3 : 3) correlated with CHD and multiple coronary artery lesions (ORs: 19.820 and 5.538, respectively, *P* < 0.05). With the carotid artery plaque-free status as a reference, the risks of CHD, severe coronary stenosis, and multiple coronary artery lesions increased 5.698-, 5.534-, and 3.215-fold, respectively—that is, from plaque-free to two plaques in carotid arteries; meanwhile, the risks of CHD and multiple coronary artery lesions increased 19.820- and 5.538-fold, respectively, that is, from plaque-free to three or more plaques in carotid arteries. In addition, the number of carotid plaques was positively correlated with the coronary Gensini score (*r* = 0.429 and *P* < 0.05); as the number of carotid plaques increased, the coronary Gensini score also increased, and the coronary artery lesions worsened.

The AUCs of carotid plaque count for predicting CHD, severe coronary stenosis, risk of coronary occlusion, single-branch coronary artery lesion, double-branch coronary artery lesion, and multiple-branch coronary artery lesion were 0.783, 0.783, 0.639, 0.615, 0.576, and 0.721, respectively. The AUCs of their predictive values, adjusted for traditional risk factors, increased to 0.901, 0.875, 0.780, 0.710, 0.702, and 0.799. All values were higher than those for the traditional risk factor model and were associated with a high predictive value. Among them, carotid plaque count predicted severe coronary artery stenosis as the highest AUC value within this prediction model, indicating that carotid plaque count was the best predictor of severe coronary artery stenosis. Therefore, carotid plaque count can be solely applied to predict CHD risk.

Carotid ultrasound has been a routine examination in daily clinical practice [22, 23]. Located in the neck, the carotid arteries are superficial and easy to observe [24]. Unlike IMT measurement, which is prone to errors, and thickness, which is affected by age and geography, carotid plaque count is a record of the number of bilateral carotid plaques. Only the plaques need to be observed and counted, and detailed observation of the plaque site, size, echo, and morphology is not required. Thus, the requirements for ultrasound machines are not too high; similarly, the requirements for ultrasound physicians or non-ultrasound physicians to perform screening are not too high. It can be easily promoted in the majority of hospitals for general public screening work. Even with no apparent clinical manifestations of CHD, such as angina pectoris, patients with early detection of carotid plaques—particularly those with three or more carotid plaques—may receive early preventive treatment, such as treatment for hypotension and hypoglycemia, lipid-lowering treatment, smoking cessation, salt restriction, body mass reduction, and exercise, to effectively reduce the incidence of acute cardiovascular and cerebrovascular lesions and mortality.

The study has some limitations. Firstly, this study is a cross-sectional study, and no causal relationship can be drawn between systemic atherosclerosis and CHD. Secondly, the population we studied was an inpatient population in a cold hospital in northern China, so the results of this study may not be applicable to other ethnic groups or the general population. Again, this study was conducted with the results of coronary angiography as an assessment of events, without a follow-up period or continued assessment of subsequent cardiovascular events, which may have led to biased results, and this discrepancy may have reduced our overall ability to observe.

## 5. Conclusion

This study shows the clinical feasibility of constructing a CHD risk prediction model by noninvasive ultrasonography of arteries (including the carotid, abdominal, and extremity arteries), combined with traditional risk factors. Specifically, the carotid artery plaque count is independently correlated with CHD risk and can be used as an independent predictor of CHD risk. The efficacy of the model for predicting CHD risk classified by carotid AS, lower limb artery AS, degree of stenosis of lower limb arteries, and the number of stenotic branches of the abdominal aortic branch arteries is large and can be used as a predictive variable for CHD risk, providing an individualized, noninvasive, simple, and easy technique for early warning, early screening, early prevention, and early intervention of clinical CHD. Abdominal aortic flow velocity and inferior mesenteric artery flow velocity are risk factors for the arterial ultrasound assessment data of CHD, and further studies are needed to explore their value.

## Figures and Tables

**Figure 1:** Arterial ultrasonography.

**Figure 2:** Correlation analysis between arterial ultrasound assessment and the coronary Gensini score. (a) Spearman correlation analysis of the carotid plaque number and the coronary artery Gensini score: correlation scatterplot; (b) Spearman correlation analysis of the lower limb plaque count and the coronary artery Gensini score: correlation scatterplot; and (c) Spearman correlation analysis of lower limb AS and the coronary artery Gensini score: correlation scatterplot.

**Figure 3:** Diagnostic value of arterial ultrasound assessment for CHD. (a) ROC curves of arterial ultrasound assessment data for CHD (before adjustment); (b) ROC curves of arterial ultrasound assessment data for severe coronary artery stenosis (before adjustment); (c) ROC curves of arterial ultrasound assessment data for coronary artery occlusion (before adjustment); (d) ROC curves of arterial ultrasound assessment data for single coronary artery lesion (before adjustment); (e) ROC curves of arterial ultrasound assessment data for double-branch coronary artery lesions (before adjustment); and (f) ROC curves of arterial ultrasound assessment data for multivessel coronary artery lesions (before adjustment).

**Figure 4:** Diagnostic efficacy of arterial ultrasound assessment combined with traditional risk factors in predicting CHD risk. (a) ROC curves of arterial ultrasound assessment data for CHD (adjustment); (b) ROC curves of arterial ultrasound assessment data for severe coronary artery stenosis (adjustment); (c) ROC curves of arterial ultrasound assessment data for coronary artery occlusion (adjustment); (d) ROC curves of arterial ultrasound assessment data for single coronary artery lesion (adjustment); (e) ROC curves of arterial ultrasound assessment data for double-branch coronary artery lesion (adjustment); and (f) ROC curves of arterial ultrasound assessment data for multivessel coronary artery lesion (adjustment).

**Table 1:** Comparison of abnormal blood biochemical indices between the CHD group and the control group.

Indicators	*n* = 343	Control group (*n* = 85)	CHD group (*n* = 258)	*χ*2	*P* value
Dyslipidemia	68.8 (236)	57.1 (48)	72.6 (188)	6.350	0.012
TC (>5.71 mmol/L)	20.7 (71)	20.2 (17)	20.8 (54)	<0.001	1.000
TG (>2.25 mmol/L)	21.9 (75)	14.3 (12)	24.3 (63)	3.180	0.075
HDL-C (<1.03 mmol/L)	35.3 (121)	22.6 (19)	39.4 (102)	7.090	0.008
LDL-C (>4.11 mmol/L)	10.2 (35)	8.3 (7)	10.8 (28)	0.198	0.657
ApoB (>1.05 g/L)	30.3 (104)	22.6 (19)	32.8 (85)	2.660	0.103
FIB(>3.5 g/L)	28.3 (97)	17.9 (15)	31.7 (82)	5.300	0.021
PLT (>300.2 × 10^9^/L)	12.2 (42)	10.7 (9)	12.7 (33)	0.091	0.763
CK-MB (>5.2 ng/ml)	21.3 (73)	1.2 (1)	27.8 (72)	25.200	<0.001
BNP (>100 pg/ml)	25.9 (89)	9.5 (8)	31.3 (81)	14.500	<0.001
hs-cTnT (>34.2 pg/ml)	44.0 (151)	8.3 (7)	55.6 (144)	55.600	<0.001
GGT (>60 U/L)	21.9 (75)	10.7 (9)	25.5 (66)	7.260	0.007
BUN (>7.1 mmol/l)	19.0 (65)	22.6 (19)	17.8 (46)	0.684	0.408
Cr (>110 umol/L)	7.3 (25)	6.0 (5)	7.7 (20)	0.090	0.764
UA (>506 umol/L)	7.0 (24)	3.6 (3)	8.1 (21)	1.370	0.242

Note: Expressed as percentages (%) (number of cases *n*).

**Table 2:** Comparison of arterial ultrasound base indicators between the CHD group and the control group.

Indicators	*n* = 363	Control group (*n* = 90)	CHD group (*n* = 273)	*t* or *w*-value	*P* value
Carotid artery internal diameter (mm)	7.9 ± 1.0	7.3 ± 1.1	8.1 ± 1.0	− 6.000	<0.001
Carotid artery IMT (mm)	0.9 ± 0.2	0.9 ± 0.2	0.9 ± 0.2	− 1.120	0.264
Vertebral artery internal diameter (mm)	3.5 ± 2.9	3.3 ± 0.4	3.6 ± 3.3	− 1.920	0.056
Vertebral artery flow velocity (cm/s)	49.9 ± 17.2	51.0 ± 10.7	49.5 ± 18.9	0.955	0.341
Subclavian artery flow velocity (cm/s)	113.1 ± 30.4	98.2 ± 29.2	118.1 ± 29.2	− 5.600	<0.001
Brachial artery internal diameter (mm)	4.7 (4.5)	4.5 (4.5)	4.7 (4.5)	3615.000	0.071
Brachial artery IMT (mm)	0.4 ± 0.1	0.3 ± 0.1	0.4 ± 0.1	− 7.340	<0.001
Abdominal aortic internal diameter (mm)	1.8 ± 0.8	1.7 ± 0.2	1.8 ± 0.9	− 2.400	0.017
Abdominal aortic flow velocity (cm/s)	79.6 ± 25.9	67.6 ± 15.8	83.5 ± 27.3	− 6.810	<0.001
Abdominal trunk flow velocity (cm/s)	161.2 ± 65.3	142.6 ± 55.9	167.3 ± 67.1	− 3.450	0.001
Superior mesenteric artery flow velocity (cm/s)	183.0 ± 62.5	160.6 ± 48.1	190.4 ± 65.0	− 4.640	<0.001
Inferior mesenteric artery flow velocity (cm/s)	144.9 ± 72.1	101.0 ± 47.9	159.4 ± 72.9	− 8.700	<0.001
Renal artery opening flow velocity (cm/s)	86.5 ± 31.8	77.2 ± 18.3	89.5 ± 34.6	− 4.330	<0.001
Renal artery opening RI	0.7 ± 0.1	0.7 ± 0.1	0.7 ± 0.1	− 4.310	<0.001
Flow velocity at the renal artery portal (cm/s)	59.4 ± 18.2	57.6 ± 16.8	60.0 ± 18.6	− 1.130	0.259
RI at renal artery portal	0.7 ± 0.1	0.6 ± 0.1	0.7 ± 0.1	− 5.070	<0.001
Femoral artery internal diameter (mm)	8.3 ± 3.1	7.9 ± 3.7	8.4 ± 2.9	− 1.090	0.278
Femoral artery IMT (mm)	0.8 ± 0.2	0.8 ± 0.2	0.8 ± 0.2	− 3.270	0.001

Note: Expressed as mean ± standard deviation (x̅±s) or with a median of M (P25, P75).

**Table 3:** Binary logistic regression analysis of arterial ultrasound base indicators and the severity of CHD lesions.

Indicators	CHD	Severe coronary artery stenosis	Coronary artery occlusion
Carotid artery internal diameter	1.609^∗^ (1.177-2.223)	1.403^∗^ (1.069-1.858)	1.069 (0.832-1.362)
Subclavian artery flow rate	1.006 (0.994-1.018)	1.006 (0.995-1.017)	0.999 (0.990-1.008)
Abdominal aortic internal diameter	1.304 (0.840-5.514)	1.231 (0.868-3.716)	1.667 (0.994-5.375)
Abdominal aortic flow velocity	1.031^∗^ (1.011-1.053)	1.016 (1.000-1.035)	1.005 (0.996-1.017)
Abdominal trunk flow velocity	0.998 (0.993-1.004)	1.001 (0.997-1.006)	1.001 (0.997-1.005)
Superior mesenteric artery flow rate	1.002 (0.996-1.009)	1.003 (0.997-1.009)	0.999 (0.994-1.003)
Inferior mesenteric artery flow velocity	1.012^∗^ (1.006-1.018)	1.010^∗^ (1.006-1.015)	1.008^∗^ (1.004-1.011)
Renal artery opening flow velocity	1.008 (0.996-1.021)	1.009(0.999-1.021)	1.003 (0.995-1.010)
Renal artery opening RI	41.638 (0.034-49491.402)	38.150 (0.068-21005.992)	9.228 (0.046-1935.147)
Renal artery portal RI	0.242 (0-324.284)	0.160 (0-104.914)	0.032 (0-10.218)

Note: Expressed as OR (95% confidence interval), ^∗^ indicates *P* < 0.05.

**Table 4:** Binary logistic regression analysis of arterial ultrasound base indicators and the number of CHD lesions.

Indicators	Single coronary artery lesion	Double coronary artery lesion	Multibranch coronary artery lesions
Carotid artery internal diameter	1.306 (0.908-1.870)	1.372^∗^ (1.015-1.871)	1.115 (0.871-1.430)
Subclavian artery flow rate	1.000 (0.986-1.013)	0.994 (0.982-1.006)	1.011^∗^ (1.002-1.020)
Abdominal aortic internal diameter	0.326 (0.057-1.101)	0.762 (0.175-1.282)	1.836 (0.986-6.311)
Abdominal aortic flow velocity	1.031^∗^ (1.010-1.054)	1.003 (0.989-1.014)	0.995 (0.982-1.005)
Abdominal trunk flow velocity	0.992^∗^ (0.984-0.999)	0.998 (0.992-1.004)	1.003 (0.999-1.008)
Superior mesenteric artery flow rate	0.997 (0.989-1.004)	1.002 (0.996-1.008)	1.001 (0.996-1.006)
Inferior mesenteric artery flow velocity	0.998 (0.992-1.003)	1.001 (0.997-1.006)	1.008^∗^ (1.004-1.012)
Renal artery opening flow velocity	1.000 (0.988-1.011)	0.996 (0.984-1.006)	1.006 (0.998-1.015)
Renal artery opening RI	0.004 (0-11.479)	0.352 (0-389.273)	85.801 (0.399-19757.822)
Renal artery portal RI	52.821 (0.013-335208.403)	12.385 (0.007-27009.612)	0.069 (0-21.913)

Note: Expressed as OR (95% confidence interval), ^∗^ indicates *P* < 0.05.

**Table 5:** Binary logistic regression analysis of ultrasound IMT thickening and plaque indicators and severity of CHD lesions.

Indicators	CHD	Severe coronary artery stenosis	Coronary artery occlusion
Brachial artery IMT	7435.122^∗^ (137.285-612104.574)	46.644^∗^ (1.857-1436.904)	3.116 (0.207-47.321)
Femoral artery IMT	0.452 (0.085-2.345)	1.041 (0.233-4.661)	1.119 (0.286-4.276)
Carotid artery plaque count			
1: 1 plaque	1.915 (0.876-4.256)	1.643 (0.792-3.430)	0.961 (0.418-2.174)
2: 2 plaques	4.121^∗^ (1.576-11.786)	6.370^∗^ (2.618-16.854)	2.710^∗^ (1.228-6.090)
3: 3 or more plaques	5.258^∗^ (2.056-14.287)	4.376^∗^ (1.990-9.895)	1.974 (0.931-4.279)
Number of subclavian artery plaques			
1: 1 plaque	0.974 (0.503-1.872)	0.786 (0.439-1.388)	0.842 (0.513-1.375)
2: 2 plaques	15701733.587 (0-NA)	26100272.902 (0-NA)	0.742 (0.094-4.294)
3: 3 or more plaques	2142739.552 (0-NA)	3620192.865 (0-NA)	0.286 (0.032-1.739)
Number of plaques in the abdominal aorta			
1: 1 plaque	4.589 (0.711-91.137)	1.719 (0.429-8.822)	0.917 (0.266-2.805)
2: 2 plaques	0.054 (0.002-1.51)	0.154 (0.006-4.099)	0 (NA-Inf)
3: 3 or more plaques	2.208 (0.959-5.448)	1.659 (0.842-3.319)	1.493 (0.873-2.552)
Number of lower-extremity-arterial plaques			
1: 1 plaque	0.233^∗^ (0.075-0.673)	0.325^∗^ (0.107-0.901)	0.526 (0.142-1.561)
2: 2 plaques	1.607(0.464-6.598)	1.327 (0.444-4.308)	0.882 (0.304-2.350)
3: 3 or more plaques	2.992^∗^ (1.237-7.807)	2.291^∗^ (1.115-4.830)	1.146 (0.637-2.059)

Note: Expressed as OR (95% confidence interval), ^∗^ indicates *P* < 0.05.

**Table 6:** Binary logistic regression analysis of ultrasound IMT thickening and plaque indicators and the number of CHD lesions.

Indicators	Single coronary artery lesion	Double coronary artery lesion	Multibranch coronary artery lesions
Brachial artery IMT	314.492^∗^ (8.134-13615.849)	75.467^∗^ (2.337-2458.444)	0.618 (0.039-10.105)
Femoral artery IMT	0.405 (0.051-2.820)	0.335 (0.045-2.227)	1.734 (0.438-6.841)
Carotid artery plaque count			
1: 1 plaque	0.817 (0.318-2.032)	1.205 (0.370-3.911)	2.449^∗^ (1.126-5.449)
2: 2 plaques	0.820 (0.297-2.161)	2.320 (0.783-7.226)	3.297^∗^ (1.465-7.614)
3: 3 or more plaques	0.283^∗^ (0.093-0.813)	1.755 (0.615-5.397)	5.680^∗^ (2.662-12.623)
Number of subclavian artery plaques			
1: 1 plaque	0.892 (0.433-1.823)	0.902 (0.467-1.740)	1.136 (0.694-1.852)
2: 2 plaques	3.573 (0.164-30.789)	3.364 (0.411-20.949)	0.518 (0.085-3.142)
3: 3 or more plaques	0 (NA-Inf)	0 (NA-Inf)	8622112.427 (0-NA)
Number of plaques in the abdominal aorta			
1: 1 plaque	1.273 (0.250-4.946)	0.761 (0.110-3.151)	1.918 (0.588-6.665)
2: 2 plaques	0 (NA-Inf)	0 (NA-Inf)	0.989 (0.035-28.170)
3: 3 or more plaques	0.739 (0.316-1.664)	1.236 (0.613-2.493)	1.495 (0.864-2.583)
Number of lower-extremity-arterial plaques			
1: 1 plaque	0 (NA-Inf)	0 (0-Inf)	1.018 (0.355-2.763)
2: 2 plaques	0.535 (0.077-2.219)	0.992 (0.209-3.488)	2.127 (0.780-5.995)
3: 3 or more plaques	0.711 (0.288-1.712)	1.216 (0.564-2.646)	1.705 (0.947-3.074)

Note: Expressed as OR (95% confidence interval), ^∗^ indicates *P* < 0.05.

**Table 7:** Binary logistic regression analysis of ultrasound stenosis indicators and the severity of CHD lesions.

Indicators	CHD	Severe coronary artery stenosis	Coronary artery occlusion
Carotid artery stenosis	0.237^∗^ (0.064-0.933)	0.366 (0.112-1.269)	0.625 (0.260-1.476)
Number of carotid artery stenosis branches			
1: 1 branch	0.427 (0.125-1.639)	0.880 (0.315-2.736)	1.048 (0.457-2.347)
2: 2 branches	3775659.253 (0-Inf)	13079803.310 (0-NA)	1.241 (0.392-3.896)
3: 3 or more branches	1845654.136 (0-NA)	5616698.794 (0-NA)	0.989 (0.156-6.210)
Degree of carotid artery stenosis			
1: <50%	3.375 (0.404-72.618)	1.549 (0.238-13.198)	1.341 (0.362-5.184)
2: 50%–69%	0.403 (0.043-4.129)	0.443 (0.052-4.416)	1.045 (0.224-4.879)
3: 70%–99%	0.353 (0.017-10.380)	0.410 (0.027-11.298)	1.880 (0.299-12.394)
4: Occlusion	0 (NA-Inf)	0 (NA-Inf)	0 (NA-Inf)
Carotid artery AS	1.222^∗^ (1.091-1.376)	1.195^∗^ (1.077-1.330)	1.033 (0.944-1.131)
Subclavian artery stenosis	1.287 (0.131-30.877)	2.020 (0.216-47.429)	0.303 (0.058-1.208)
Classification of the number of stenotic branches in the carotid vessels			
1: 1 branch	1.150 (0.364-4.379)	1.738 (0.558-6.553)	0.883 (0.302-2.360)
2: 2 branches	2.559 (0.297-65.019)	4.578 (0.560-109.759)	0.463 (0.089-2.043)
3: 3 or more branches	26248622924236.600 (0-NA)	Inf (0-NA)	0.293 (0.043-1.733)
Stenosis of the abdominal trunk	1.306 (0.652-2.706)	1.848 (0.961-3.668)	1.770^∗^ (1.031-3.033)
Superior mesenteric artery stenosis	4.317 (0.776-81.153)	2.974 (0.737-20.118)	0.538 (0.215-1.267)
Number of stenotic branches of abdominal aortic branch arteries			
1: 1 branch	1.295 (0.707-2.448)	1.701 (0.955-3.104)	1.294 (0.749-2.211)
2: 2 branches	25074606.442 (0-NA)	40965865.805 (0-NA)	2.162 (0.903-5.261)
3: 3 or more branches	13563499.532 (0-NA)	21583085.963 (0-NA)	0.265 (0.013-1.959)
Lower-extremity-artery stenosis	0.972 (0.219-5.374)	1.159 (0.328-4.595)	1.327 (0.572-3.036)
Number of lower-extremity-artery stenosis			
1: 1 branch	4.093 (1.114-26.565)	5.832^∗^ (1.602-37.542)	1.724 (0.651-4.329)
2: 2 branches	52135861.337 (0-Inf)	11.047^∗^ (3.178-70.049)	2.764^∗^ (1.323-5.801)
3: 3 or more branches	12.231^∗^ (2.312-230.777)	15.937^∗^ (3.149-292.109)	5.736^∗^ (2.492-14.081)
Degree of stenosis of lower-extremity arteries			
1: 30%–49%	2.958 (0.491-56.476)	4.301 (0.71-82.253)	0 (NA-Inf)
2: 50–75%	7.078 (1.385-129.410)	10.572^∗^ (2.066-193.348)	2.879^∗^ (1.091-7.729)
3: >75%	40265607.462 (0-NA)	59063290.83 (0-NA)	3.749^∗^(1.348-11.047)
4: Occlusion	19.585^∗^(4.118-351.031)	8.958^∗^(3.112-37.903)	3.287^∗^ (1.739-6.296)
Lower-extremity-artery AS	1.212^∗^ (1.098-1.352)	1.170^∗^ (1.075-1.28)	1.055^∗^ (1.008-1.107)

**Table 8:** Binary logistic regression analysis of ultrasound stenosis indicators and the number of CHD lesions.

Indicators	Single coronary artery lesion	Double coronary artery lesion	Multibranch coronary artery lesions
Carotid artery stenosis	1.551 (0.287-6.652)	0.676 (0.218-1.971)	0.310^∗^ (0.123-0.768)
Number of carotid artery stenosis branches			
1: 1 branch	1.144 (0.245-3.993)	0.858 (0.261-2.397)	0.712 (0.312-1.644)
2: 2 branches	0 (0-Inf)	0.692 (0.100-2.947)	2.570 (0.623-17.549)
3: 3 or more branches	0 (NA-Inf)	3.797 (0.389-37.882)	0.372 (0.042-3.326)
Degree of carotid artery stenosis			
1: <50%	2.384 (0.328-21.347)	1.954 (0.326-15.871)	0.618 (0.158-2.371)
2: 50%–69%	0 (NA-Inf)	1.136 (0.102-12.163)	0.699 (0.134-3.821)
3: 70%–99%	0 (NA-Inf)	0.695 (0.026-10.195)	0.909 (0.123-8.563)
4: Occlusion	0 (NA-Inf)	0 (NA-Inf)	0.955 (0.030-29.247)
Carotid artery AS	0.884 (0.773-1.005)	1.118 (0.997-1.257)	1.199^∗^ (1.093-1.319)
Subclavian artery stenosis	1.336 (0.065-9.777)	0.330 (0.017-2.046)	1.027 (0.201-6.310)
Classification of the number of stenotic branches in the carotid vessels			
1: 1 branch	0.906 (0.138-3.476)	0.616 (0.091-2.391)	1.545 (0.567-4.332)
2: 2 branches	0 (0-Inf)	1.213 (0.120-7.785)	2.412 (0.518-12.701)
3: 3 or more branches	0 (0-Inf)	2.766 (0.212-29.395)	2.239 (0.339-17.027)
Stenosis of the abdominal trunk	0.384 (0.125-0.958)	1.029 (0.493-2.048)	1.720 (0.982-3.02)
Superior mesenteric artery stenosis	0.900 (0.133-3.637)	0.850 (0.254-2.418)	1.660 (0.651-4.496)
Number of stenotic branches of abdominal aortic branch arteries			
1: 1 branch	0.507 (0.198-1.133)	1.208 (0.601-2.331)	1.489 (0.877-2.525)
2: 2 branches	0.306 (0.017-1.596)	0.482 (0.074-1.78)	8.282^∗^ (2.639-36.593)
3: 3 or more branches	0 (NA-Inf)	1.202 (0.060-8.376)	3.197 (0.432-66.126)
Lower-extremity-artery stenosis	0.340 (0.057-1.585)	0.727 (0.226-2.184)	1.733 (0.694-4.411)
Number of lower-extremity-artery stenosis			
1: 1 branch	0.299 (0.016-1.544)	0.472 (0.068-1.866)	5.303^∗^ (1.976-16.831)
2: 2 branches	0.350 (0.054-1.255)	2.109 (0.862-4.843)	3.233^∗^ (1.537-7.124)
3: 3 or more branches	0.201 (0.011-1.09)	0.241 (0.032-1.032)	11.817^∗^ (4.183-43.102)
Degree of stenosis of lower-extremity arteries			
1: 30%–49%	0.952 (0.049-5.94)	0.775 (0.040-4.668)	2.605 (0.597-13.241)
2: 50%–75%	0 (NA-Inf)	1.151 (0.256-3.742)	5.421^∗^ (1.839-19.809)
3: >75%	0 (NA-Inf)	0.829 (0.126-3.169)	10.895^∗^ (2.898-70.983)
4: Occlusion	0.421 (0.098-1.253)	1.119 (0.448-2.530)	4.511^∗^ (2.256-9.565)
Lower-extremity-artery AS	1.008 (0.922-1.093)	1.005 (0.945-1.065)	1.059 (1.002-1.123)

**Table 9:** Spearman or Pearson correlation analysis between the arterial ultrasound data and the coronary artery Gensini score.

Indicator	Correlation factor	*Pvalue*
Carotid IMT	0.089	0.103
Brachial artery IMT	0.250	<0.001
Femoral artery IMT	0.215	<0.001
Carotid artery plaque count	0.429	<0.001
Subclavian artery plaque count	0.126	0.016
Abdominal aortic flow velocity	0.092	0.081
Inferior mesenteric artery flow rate	0.348	<0.001
Abdominal aortic plaque	0.313	<0.001
Lower-extremity-artery plaque	0.408	<0.001
Carotid artery AS	0.319	<0.001
Lower-extremity-artery AS	0.397	<0.001
Degree of carotid stenosis	0.192	<0.001
Classification of carotid artery stenosis branch number	0.200	<0.001
Classification of the number of stenotic branches in the carotid vessels	0.202	<0.001
Number of stenotic branches of abdominal aortic branch arteries	0.285	<0.001
Lower-extremity-artery stenosis branch number classification	0.375	<0.001
Degree of stenosis of lower-extremity arteries	0.367	<0.001

**Table 10:** Area under the curve of the diagnostic value of the arterial ultrasound evaluation data for the severity of CHD lesions (before adjustment).

Indicators	CHD	Coronary artery severe stenosis	Coronary artery occlusion
	AUC (95% confidence interval)	AUC (95% confidence interval)	AUC (95% confidence interval)
Carotid artery plaque count	0.783 (0.733-0.833)	0.783 (0.735-0.831)	0.639 (0.578-0.700)
Carotid artery AS	0.750 (0.687-0.814)	0.695 (0.633-0.757)	0.608 (0.548-0.669)
Inferior mesenteric artery flow velocity	0.738 (0.677-0.800)	0.732 (0.676-0.789)	0.585 (0.524-0.647)
Abdominal aortic flow velocity	0.749 (0.691-0.808)	0.733 (0.678-0.789)	0.668 (0.611-0.726)
Number of abdominal aortic plaques	0.690 (0.643-0.737)	0.662 (0.613-0.711)	0.595 (0.540-0.650)
Number of stenotic branches of abdominal aortic branch arteries	0.758 (0.700-0.815)	0.739 (0.684-0.795)	0.614 (0.556-0.672)
Lower-extremity-artery plaque count	0.600 (0.551-0.650)	0.627 (0.581-0.672)	0.581 (0.527-0.636)
Lower-extremity-artery stenosis classification	0.734 (0.683-0.784)	0.711 (0.661-0.762)	0.584 (0.527-0.641)
Degree of stenosis of lower-extremity arteries	0.653 (0.620-0.686)	0.662 (0.626-0.697)	0.614 (0.562-0.666)
Lower-extremity-artery AS	0.652 (0.619-0.686)	0.662 (0.626-0.697)	0.635 (0.585-0.686)

**Table 11:** Area under the curve of diagnostic value of arterial ultrasound evaluation data for number of coronary artery lesions (before adjustment).

Indicators	Single coronary artery lesion	Double coronary artery lesion	Multi-branch coronary artery lesions
	AUC (95% confidence interval)	AUC (95% confidence interval)	AUC (95% confidence interval)
Carotid artery plaque count	0.615 (0.536-0.693)	0.576 (0.502-0.650)	0.721 (0.670-0.773)
Carotid artery AS	0.611 (0.532-0.691)	0.563 (0.484-0.643)	0.599 (0.540-0.658)
Inferior mesenteric artery flow velocity	0.645 (0.566-0.724)	0.560 (0.480-0.640)	0.711 (0.658-0.765)
Abdominal aortic flow velocity	0.578 (0.494-0.662)	0.540 (0.463-0.617)	0.698 (0.644-0.753)
Number of abdominal aortic plaques	0.577 (0.504-0.649)	0.582 (0.507-0.657)	0.625 (0.574-0.676)
Number of stenotic branches of abdominal aortic branch arteries	0.642 (0.563-0.720)	0.593 (0.517-0.668)	0.714 (0.663-0.765)
Lower-extremity-artery plaque count	0.601 (0.542-0.660)	0.537 (0.467-0.607)	0.621 (0.572-0.670)
Classification of lower-extremity-artery stenosis	0.614 (0.542-0.686)	0.601 (0.530-0.672)	0.650 (0.598-0.703)
Degree of stenosis of lower-extremity arteries	0.605 (0.558-0.652)	0.595 (0.531-0.658)	0.663 (0.619-0.707)
Lower-extremity-artery AS	0.608 (0.564-0.652)	0.515 (0.448-0.581)	0.659 (0.615-0.704)

**Table 12:** Logistic regression analysis of arterial ultrasound assessment data with the risk of CHD, severe coronary artery stenosis, and coronary artery occlusion (adjusted).

Indicator	CHD	Severe coronary artery stenosis	Coronary artery occlusion
Gender (male)	1.497 (0.569-3.964)	1.137 (0.519-2.475)	1.590 (0.841-3.036)
Age	1.015 (0.964-1.072)	0.977 (0.937-1.018)	0.976 (0.943-1.009)
History of diabetes	0.958 (0.374-2.493)	1.599 (0.735-3.567)	1.507 (0.832-2.720)
History of hypertension	1.526 (0.646-3.624)	1.408 (0.695-2.852)	0.887 (0.487-1.621)
History of smoking	1.069 (0.375-2.939)	1.041 (0.444-2.395)	0.913 (0.474-1.750)
High-salt diet	2.235 (0.967-5.290)	1.383 (0.675-2.827)	0.759 (0.413-1.391)
HDL-C abnormalities	1.481 (0.596-3.760)	1.352 (0.665-2.772)	2.282^∗^ (1.305-4.034)
CK.MB	18.587^∗^ (2.508-413.663)	1.969 (0.663-6.338)	2.896^∗^ (1.429-5.977)
BNP	1.538 (0.523-4.881)	1.166 (0.501-2.779)	2.212^∗^ (1.194-4.118)
Hs-cTnI	7.161^∗^ (2.458-24.113)	5.673^∗^ (2.519-13.607)	1.609 (0.853-3.031)
GGT abnormality	2.779 (0.926-9.329)	1.016 (0.449-2.352)	1.540 (0.810-2.921)
Carotid plaque count			
1: 1 plaque	2.805 (0.800-10.027)	1.292 (0.451-3.617)	0.687 (0.252-1.827)
2: 2 plaques	5.698^∗^ (1.049-31.231)	5.534^∗^ (1.348-22.227)	2.676 (0.911-8.073)
3: 3 or more plaques	19.820^∗^ (1.963-210.376)	5.839 (0.863-35.828)	2.541 (0.681-10.023)
Carotid AS	0.797 (0.605-1.070)	0.926 (0.749-1.183)	0.891 (0.760-1.030)
Number of abdominal aortic plaques			
1: 1 plaque	0.780 (0.091-17.130)	0.489 (0.090-3.155)	0.274 (0.047-1.237)
2: 2 plaques	0.062 (0.002-2.463)	0.105 (0.003-3.736)	0 (NA-Inf)
3: 3 or more plaques	1.126 (0.365-3.558)	0.870 (0.370-2.029)	1.134 (0.602-2.126)
Abdominal aortic flow velocity	1.061^∗^ (1.032-1.095)	1.027^∗^ (1.005-1.051)	1.000 (0.986-1.010)
Inferior mesenteric artery flow velocity	0.997 (0.989-1.006)	1.002 (0.996-1.008)	1.005^∗^ (1.000-1.009)
Number of stenotic branches of abdominal aortic branch arteries			
1: 1 branch	1.038 (0.458-2.366)	1.528 (0.756-3.141)	1.335 (0.712-2.487)
2: 2 branches	16177120.935 (0-Inf)	27977008.025 (0-Inf)	2.204 (0.804-6.224)
3: 3 or more branches	3651475.546 (0-NA)	7389775.573 (0-NA)	0.221 (0.010-1.710)
Lower-extremity-arterial plaque count			
1: 1 plaque	0.186^∗^ (0.042-0.740)	0.230^∗^ (0.059-0.815)	0.529 (0.129-1.774)
2: 2 plaques	1.732 (0.279-12.497)	0.756 (0.171-3.524)	0.969 (0.283-3.126)
3: 3 or more plaques	0.458 (0.043-4.184)	0.203 (0.033-1.119)	0.512 (0.195-1.291)
Number of arterial stenosis in the lower extremity			
1: 1 branch	0.377 (0.036-5.493)	1.154 (0.163-13.369)	0.871 (0.249-2.925)
2: 2 branches	419456.688 (0-Inf)	0.178 (0.015-2.459)	1.312 (0.359-4.719)
3: 3 and more than 3 branches	0.007 (0-2.006)	0.025 (0.001-1.679)	2.168 (0.259-19.413)
Degree of arterial stenosis in the lower limbs			
1: 30%–49%	0.388 (0.036-9.235)	1.372 (0.161-30.973)	0 (NA-Inf)
2: 50%–75%	2.059 (0.261-45.416)	4.435 (0.673-90.231)	1.803 (0.581-5.768)
3: >75%	11955619.905 (0-NA)	24183018.001 (0-NA)	2.660 (0.751-10.068)
4: Occlusion	8.860^∗^ (1.537-169.202)	4.907^∗^ (1.448-22.851)	2.920^∗^ (1.335-6.503)
Lower-extremity-artery AS	1.376^∗^ (1.044-1.881)	1.409^∗^ (1.125-1.807)	1.046 (0.947-1.160)

## Data Availability

No data were used to support this study.
